RETRACTED

# Do Chinese children need parental supervision to manage their out-of-school visual art activities and academic work time?

**DOI:** 10.3389/fpsyg.2022.987644

**Published:** 2022-09-14

**Authors:** Endale Tadesse, Sabika Khalid, Chunhai Gao, Moges Assefa Legese

**Affiliations:** ^1^College of Teacher Education, Zhejiang Normal University, Jinhua, China; ^2^Faculty of Education, Shenzhen University, Shenzhen, China; ^3^School of Business, Hohai University, Nanjing, China

**Keywords:** visual art, extracurricular activities, art interest, parental support, socioeconomic status, academic performance

## Abstract

Unlike in Western countries, scholars and the Chinese government pay less attention to the role of extracurricular activities (ECAs) in fostering children’s cognitive and non-cognitive well-being. Accordingly, essential ECAs such as visual arts programs are serviced by expensive privately owned schools, creating social injustice. The primary aim of the current study is to examine whether children benefit from ECAs if parental support and guidance for managing time spent on ECAs and academics exist based on the threshold model. The study comprised over 2,400 primary school students in one Chinese province and considered the SES of the area. Surprisingly, the present study’s findings illustrate that contemporary Chinese parents differ from traditionally aggressive and overbearing parents who do not value their children’s interests. However, the current study finding suggested that children’s participation in out-of-school visual art activities doesn’t have a substantial value in promoting children’s academic performance in the face of genuine interest and supportive parenting, which negates the threshold model.

## Introduction

Due to the extensive application of in-school and out-of-school extracurricular activities (ECAs) for children’s cognitive and non-cognitive development in Western countries (Marsh and Kleitman, 2002; Covay and Carbonaro, 2010; Kadar-Satat, 2015; Mansour et al., 2016), in recent years, the Chinese government has called for a society in which children and adolescents cherish and celebrate ECAs in and out of school (Ren et al., 2020), especially visual art education (Law and Ho, 2011; Lockette, 2012; Hui et al., 2015; Zhang and Tang, 2017; Chiu and Lau, 2018; Ye, 2018). However, as is well-documented in other countries (e.g., Mansour, 2013; Jindal-Snape et al., 2018; Morris, 2018), in China, in-school visual art education and other ECAs possess low resources and incompetent teachers that repress children’s creativity and innovation (c.f. Lowry and Wolf, 1988; Choi et al., 2005; Ho, 2011; Jolley and Zhang, 2012; Lockette, 2012; Jin, 2017), as reflected by consecutive PISA results (Jin, 2017; Zhang and Tang, 2017). Although in-school ECAs do not receive the necessary attention from the government, their effects surpass those of out-of-school ECAs (Marsh and Kleitman, 2002). However, this exceptional reality exists for the developed countries that promote ECAs. A mixed method study in China surveying parental attitudes found that parents witnessed and observed their children’s activities outside school (Lau and Cheng, 2016). Additionally, in the past decade, traditional Chinese schools have taught visual arts to children by copying an existing painting or drawing, which creates creativity disparities across China and Western countries (Lowry and Wolf, 1988; Piscitelli et al., 1999; Jolley and Zhang, 2012; Lockette, 2012), and by contemplating Confucian teachings (Zhang and Tang, 2017; Chiu and Lau, 2018; Ye, 2018) and rote learning (Law and Ho, 2011; Ho et al., 2017; Jin, 2017). Thus, parents who sincerely seek to engage their children in multiple ECAs enroll them in expensive private institutions (Choi et al., 2005; Lau and Cheng, 2016; Zhang and Tang, 2017; Chiu and Lau, 2018; Li and Qiu, 2018; Ye, 2018; Qurban et al., 2019; Liu et al., 2020; Kong, 2021). Chinese parents primarily involve their children in sports (Qurban et al., 2019), music lessons (e.g., Choi et al., 2005; Ho, 2011; Law and Ho, 2011; Kong, 2021), STEM and language ECAs (Lau and Cheng, 2016; Zhang and Tang, 2017). Unfortunately, scholars have been unable to determine the causal effect of out-of-school visual art participation on children’s in-school learning outcomes due to their narrow research scope (Hui et al., 2015; Foster and Marcus Jenkins, 2017; Ren et al., 2020).

RETRACTED

To the best of our knowledge, the present study considered three issues previously unconsidered in Chinese or foreign research. First, surprisingly, scholars in China have given very little attention to the implications of visual art education for children’s non-cognitive skills (self-esteem, self-efficacy, peer communication, creativity, and emotion) and cognitive skills (academic performance or learning outcomes). In fact, national and international literature regarding the application of ECAs to children’s development is dominated by music, sport, dancing, and STEM-oriented activities. For instance, Jindal-Snape and their colleagues conducted a systematic review to fuse the literature on out-of-school visual art activities, although they found fewer than five relevant studies, and most studies considered music as a representative ECA (Jindal-Snape et al., 2018). Hence, this paper aims to examine the extent children’s visual art participation could leverage academic performance; Second, although there are emerging studies in China that assess the significance of different ECAs, much of this evidence is from research conducted in Hong Kong (e.g., Choi et al., 2005; Ho, 2011; Hui et al., 2015; Lau and Cheng, 2016; Chiu and Lau, 2018), Shanghai and Beijing (Ren et al., 2020; Kong, 2021). These cities are highly economically and culturally developed; the children in these cities can choose the activities they prefer, and there are minor economic disparities that prevent parents from having the financial resources to send their children to ECAs (Choi et al., 2005; Ho, 2011; Lau and Cheng, 2016; Chiu and Lau, 2018; Poon, 2020). For instance, 77% of preschool children in Hong Kong participate in various ECAs, which are expensive (Ren et al., 2020), revealing the role of social class and parental support (Kong, 2021). Thus, the current study considered an economically distributed setting to explore the association between parental cultural capital, parental support, and the likelihood of participating in visual art activities offered by private training centers. In a nutshell, to the best of our knowledge, this is the first national and international level evidence that possesses an overall purpose to assess the impact of parental socioeconomic (SES) on student academic performance by considering children’s visual art interest, parental support, and out-of-school visual art participation. Many studies on parental support in China have extensively focused on music and second-language ECAs (e.g., Choi et al., 2005; Ho, 2011; Law and Ho, 2011; Chiu and Lau, 2018; Jindal-Snape et al., 2018; Qurban et al., 2019; Kong, 2021), which are deemed incompatible with the current educational goals of China. Additionally, those studies that consider parental support of ECAs as a moderator (Chiu and Lau, 2018; Ren et al., 2020) assume children’s interests and financial capacity to mediate this relationship. Hence, this paper makes a substantial contribution to the national and international literature and has implications for Chinese government policy-makers and society by explaining the tangible, robust evidence regarding visual art education, which is the contemporary focal point and prevalent cultural activity in the Chinese community.

RETRACTED

## Literature review

### Extracurricular participation of children based on child interest and parental support

Worldwide, it is believed that parental support is the frontline agency children need to participate in ECAs (Anderson et al., 2003; Dumais, 2006; Mansour et al., 2016; Morris, 2018). Although the literature on the application of extracurricular activities in China has concentrated on China’s most culturally, parenting-extensive, and economically internationalized cities, we recap the diverse literature reflecting various aspects related to the effects of ECAs. Chinese parents are well-known for “tiger parenting,” which values children’s high academic achievements, given that China is a meritocratic county (Choi et al., 2005; Ho, 2011; Lau and Cheng, 2016; Chiu and Lau, 2018, p. 478; Poon, 2020) with limited family size (Piscitelli et al., 1999; Ren et al., 2020). Unlike Western children, Chinese children do not have the gumption or confidence to question their parents; instead, they are obedient and humble regarding directions given by their family (Lockette, 2012; Ho et al., 2017; Chiu and Lau, 2018; Qurban et al., 2019; Kong, 2021). Consequently, parents exhibit aggressive parental control or supervise their children to ensure they do whatever it takes to be competitive (Lowry and Wolf, 1988). A previous study that involved ECA teachers, artists, and researchers in this area claimed that Chinese children participate in ECAs for the primary purpose of skill building, while Western countries use these activities to increase children’s appreciation of their skills and discover themselves (Lowry and Wolf, 1988; Smith and Smith, 2008). However, additional evidence in contemporary China negates this view (Choi et al., 2005; Ho. 2011). Indeed, the parental support perceived by children significantly contributes to the interest they have in an activity (Anderson et al., 2003). Chinese parents with high cultural capital are generally busy with their professional duties, making them incapable of being involved in their children’s ECAs, which diminishes the significance of ECA participation (Ho, 2011). A piece of recent evidence echoed this argument by showing the substantial worth of parental time investment in magnifying the benefit of visual art activities regardless of financial investment (Gao et al., 2022).

In doing so, it is crucial to investigate ECAs independently in the era of Chinese children extensively participating in several ECAs. Studies have noted that in the Chinese cultural tradition of parenting, the mother has considerable autonomy in deciding the types of extracurricular activities children engage in Lau and Cheng (2016), Zhang and Tang (2017), Chiu and Lau (2018), Kong (2021), and the father determines whether disciplinary action is needed for poor in- and out-of-school performance (Lowry and Wolf, 1988). Accordingly, recent evidence from Hong Kong illustrates that children cannot obtain the benefits of ECAs when their activities are overscheduled by several ECAs, which makes them fatigued than cherishing (Chiu and Lau, 2018), although a previous study assumes that the more ECAs children engage in, the greater their development (Dumais, 2006).

RETRACTED

Extracurricular activities are universally recognized and acknowledged human activities, but this does not mean anyone can participate in an ECA without being interested in it (McManus and Furnham, 2006). Plausibly, a study in the United States found that children lose interest in ECAs when their parents exercise pressure and controlling behavior (Anderson et al., 2003). We speculate that Chinese parents use strict supervision to control the time their children devote to ECAs to prevent it from damaging their academic performance. In addition, children who understand the value of their academic performance for their future lives manage the time they engage in ECAs (Mansour et al., 2016). Otherwise, children will not develop through the activities, and parental financial, time and energy investments are useless (Anderson et al., 2003). Based on the existing literature, the current study speculates the following assumptions.

*H*_1_ *: The active participation of children in visual art ECAs is determined by their interests.*

*H*_2_ *: The association between children’s art interest and active participation in visual art ECAs is mediated by parental support.*

### Visual art activities and academic performance

Out-of-school ECAs are general claimed to play a significant role in assuring dimensions of children’s well-being, such as social competency, life satisfaction, and academic performance (Dumais, 2006; Ho, 2011; Lau and Cheng, 2016), even though they have been found to have null (Marsh and Kleitman, 2002; Foster and Marcus Jenkins, 2017) or moderate (Dumais, 2006; Covay and Carbonaro, 2010) effects on children’s academic development. Interestingly, a famous scholar in this area used a more rigorous and causal research method to confirm that the influence of out-of-school ECAs on student school-related performance is lower than that of in-school ECAs (Marsh and Kleitman, 2002). Therefore, ECAs have promising prospects since they engage children in exciting activities that boost their communication with peers, positive emotions, aesthetic cognition, and responsibility, which have strong links with school academic performance (Dumais, 2006; Ho, 2011; Lau and Cheng, 2016; Morris, 2018; Kong, 2021). Moreover, visual arts are not comparable to other ECAs since they require genuine and persistent interest (Lowry and Wolf, 1988). However, empirical evidence strongly supports that such intended outcomes can be obtained as long as children have a definite interest in the specific activity and genuine support from their parents (Zhang and Tang, 2017; Qurban et al., 2019). In addition, another study indicates that children need to participate in a limited number of ECAs in which they are interested in avoiding affecting their academic performance (Lau and Cheng, 2016). Nevertheless, a recent longitudinal survey in Shanghai emphasized that children engaged in ECAs exhibit a radical improvement in math and social skills. However, unconstrained and unmanaged investment in ECAs, the benefit to zero in the limit since money cannot buy everything (Ren et al., 2020). Therefore, in addition to financial investment, parents must devote their time to supporting and overseeing their children’s ECA participation to obtain the intended benefits (Dumais, 2006; Ho, 2011; Kong, 2021), including parent-child attachment (Ho, 2011).

RETRACTED

Thus, considering the literature gaps, the current study targeted primary school-aged children who participated in any ECA based on their interests, choices, and parental guidance. This study investigates what enhances children’s ECA participation and improves academic performance. The growing volume of studies on children’s interest in out-of-school ECAs has shown boys prefer activities that are not *girly* but entail physical exercise, such as sports, dancing, and music, while girls cherish visual arts, music, and theater (Anderson et al., 2003; McManus and Furnham, 2006; Smith and Smith, 2008; Mansour et al., 2016; Ye, 2018; Qurban et al., 2019; Kong, 2021). Additionally, children lose interest in ECAs over time and in adolescence (Smith and Smith, 2008; Mansour et al., 2016; Foster and Marcus Jenkins, 2017; Jindal-Snape et al., 2018; Morris, 2018; Ye, 2018); however, a longitudinal study of senior high school students found a substantial effect of ECAs on students’ learning attainment (Marsh and Kleitman, 2002).

Compared with other ECAs, visual art education plays a vital role in Chinese children’s cognitive development (Jolley and Zhang, 2012). During visual art participation, children start fostering their ability to explain their emotions, which Chinese culture limits (Dumais, 2006; Ho et al., 2017); building the confidence to share their work with others; developing communication skills with peers; and obtaining solid self-efficacy in appraising the work of others (Marsh and Kleitman, 2002; Jolley and Zhang, 2012; Ho et al., 2017; Morris, 2018). Previous research has found that students with high academic achievement are interested in and participate in visual art activities in and out of school (Mansour et al., 2016).

Due to the noteworthy role of art in children’s learning engagement, the twenty first-century core curriculum should include art. This integration of art into education has brought substantial attention to teaching practices and lifelong student learning, albeit visual art is more valuable when given separately (Hui et al., 2015). In addition, ECAs such as sports have a constricted likelihood of fostering children’s self-esteem and school academic attainment (Qurban et al., 2019). Likewise, a recent systematic review that synthesized 24 studies from Western countries argued that the anticipated effect of visual art activities becomes uncertain when schools integrate them with other subjects or ECAs such as sports (Jindal-Snape et al., 2018).

RETRACTED

These fundamental skills, which can rarely be obtained from other ECAs, are strongly related to a child’s refreshed and polished mind that enjoys in-school tasks (Morris, 2018). Chinese art education has traditionally promoted art values and pedagogical practices different from Western art education (Kong, 2021). Chinese art in its various forms (e.g., drawing, painting, and calligraphy) has had enduring value in Chinese culture (Jolley and Zhang, 2012). In the contemporary world, parents who can yield decent cultural capital send their children to out-of-school art schools that are well-resourced and possess professional teachers to cultivate solid creativity and facilitate social, psychological, and academic adjustments in their children (Piscitelli et al., 1999; Dumais, 2006; Smith and Smith, 2008; Hui et al., 2015; Foster and Marcus Jenkins, 2017; Chiu and Lau, 2018; Ye, 2018; Ren et al., 2020). The results of a quasi-experimental study on seven kindergartens conducting art projects designed by Hong Kong officials indicate that children who acquire art education solely through professional art teachers exhibit pronounced development in verbal and figural creativity (Hui et al., 2015). A similar finding was obtained in the United Kingdom (Kadar-Satat, 2015). Based on the consistent evidence discussed above, the present study proposes the following hypothesis:

*H3: Children’s active participation in visual art activities substantially impacts their academic performance.*

### Extracurricular activities and socioeconomic status

A large volume of Western literature stresses the substantial impact of socioeconomic status (SES) on the cultural capital advantage children obtain from, e.g., ECAs (e.g., Anderson et al., 2003; Covay and Carbonaro, 2010; Kadar-Satat, 2015; Mansour et al., 2016; Foster and Marcus Jenkins, 2017; Morris, 2018). Unsurprisingly, a large body of evidence supports the extent to which parent SES determines children’s academic performance (Liu et al., 2020), particularly in math (Covay and Carbonaro, 2010), although the association is indirect (Anderson et al., 2003; Mansour et al., 2016; Li and Qiu, 2018; Poon, 2020). Parents with a steady income can afford to meet their children’s academic and non-academic resource needs, which undoubtedly impacts their academic performance (Covay and Carbonaro, 2010; Foster and Marcus Jenkins, 2017; Zhang and Tang, 2017; Jindal-Snape et al., 2018; Ye, 2018; Ren et al., 2020); furthermore, recent research has found that high-SES parents rigorously support and have high expectations of their children to utilize the cultural capital they possess (Poon, 2020). Surprisingly, Poon’s structural equation model (SEM) article shows that low-income Chinese parents do not have time for their children given that they have more than one job, which results in low support for and expectations regarding their children’s academic and non-academic activities (Poon, 2020). That allows low-SES children to spend their leisure time in any activities they choose, regardless of whether they impact their development (Dumais, 2006). Apart from formal out-of-school visual art classes, parents should dedicate time with their children to art exhibitions and museums to promote the art emotion, cognition, and self-efficacy crucial for a child’s in-school learning motivation and achievement (Morris, 2018).

RETRACTED

Indeed, a recent report claimed that student academic outcomes are the primary indicator of a country’s education equality and equity (OECD, 2016; Li and Qiu, 2018). The 2015 Programme for International Student Assessment (PISA) results showed that 18% of the academic performance of the students from Chinese who responded to the assessment was explained by their parental SES (OECD, 2016), which was lower than the rate in another study (Li and Qiu, 2018; Ye, 2018). Indeed, only four of the 36 provinces participated in the assessment (Liu et al., 2020). A subsequent survey study of 25 provincial households revealed family SES strongly predicts children’s learning performance (Li and Qiu, 2018). Nonetheless, a recent meta-analysis in six regions of China obtained the exciting finding that the relationship between SES and student academic attainment weakens over the years (Liu et al., 2020), although another study revealed growth in inequality income (Liu et al., 2020; Ren et al., 2020). Liu et al. (2020) urge further investigation to understand the potential mediators and moderators of the impact of socioeconomic status on student academic performance in more economically well-off provinces. Hence, in the era of free compulsory education, children attend school without parental monetary strain, yet academic achievement and success are still predicted by SES (Li and Qiu, 2018; Liu et al., 2020). Nevertheless, out-of-school ECAs such as visual arts increase the effect of SES on children’s learning outcomes (Zhang and Tang, 2017; Ye, 2018; Ren et al., 2020; Gao et al., 2022). Such a claim was also made by international studies that also found a strong bond between parental financial and educational stability with children’s participation in ECAs (McManus and Furnham, 2006; Covay and Carbonaro, 2010; Kadar-Satat, 2015; Mansour et al., 2016; Foster and Marcus Jenkins, 2017; Morris, 2018). The results of Covay and Carbonaro’s (2010) hierarchal model postulate that the causal relationship between SES and learning outcomes is mediated by participation in ECAs. Then, Mansour et al. (2016) claimed parent SES levels impact children’s out-of-school art participation, and this relationship is mainly affected by parental education level.

RETRACTED

Accordingly, children from affluent parents are more likely to participate in out-of-school ECAs and receive family involvement in or out of the home to strengthen their ability to participate (Ho, 2011; Ye, 2018; Qurban et al., 2019; Kong, 2021). The study of Ye in Shanghai examined high school participation in ECAs and found that although SES determines the tendency of adolescents to engage in out-of-school ECAs, parents’ educational level and occupation cannot determine the frequency at which their children visit ECA centers since adolescents experience peer pressure that outweighs parental participation (Ye, 2018). Alternatively, parents withdraw their children from ECAs they are interested in so that they can focus on the university entrance examination that predicts their future life paths (Choi et al., 2005; Ho, 2011; Mansour et al., 2016; Qurban et al., 2019); therefore, ECAs are a means of laying a foundation for future learning competency (Chiu and Lau, 2018). Furthermore, a recent study in the same city found that children from low-SES families benefit more from ECAs than their high-SES counterparts since low-SES children effectively use ECAs that cannot be easily accessed at home (Ren et al., 2020), and an American study found the same (Marsh and Kleitman, 2002; Dumais, 2006; Covay and Carbonaro, 2010). Accordingly, the following hypotheses are posited:

*H*_4_ *: Parental socioeconomic status directly impacts their children’s academic performance.*

*H*_5_ *: The relationship between parental socioeconomic status and academic performance is mediated by art interest, parental support, and visual art participation.*

*H*_6_ *: Art interest, parental support, and visual art participation play a serial mediating role in the relationship between parental socioeconomic status and academic performance.*

RETRACTED

### Theoretical framework

What do we mean by cultural capital? In 1973, the famous scholar Bourdieu theorized that cultural capital is mainly exhibited by a personal inclination toward social class-specific lifestyles instilled through prolonged socialization within the family (Bourdieu, 1973). Thus, the consequence of the different socialization experienced by children at various socioeconomic levels is a class-based habitus conveyed by a certain level of cultural capital (Bourdieu, 1973; Dumais, 2006; Smith and Smith, 2008; Kadar-Satat, 2015). Participating in ECAs, such as visual art education out of school, is a type of cultural activity that sets the social activity boundary for middle and lower social class individuals who are academically advanced and have low incomes (Poon, 2020). Furthermore, cultural capital expresses individuals’ social class and actively reproduces social and educational inequality (Covay and Carbonaro, 2010; Kadar-Satat, 2015; Foster and Marcus Jenkins, 2017; Kong, 2021). This theory is essential for investigating the direct relationship between participation in ECAs and SES (Kadar-Satat, 2015) since assessing the association at the general level is problematic without considering latent variables (Dumais, 2006). A review paper criticized scholars for using sloppy research methods and findings due to being unaware of the theory supporting visual art activities (Jindal-Snape et al., 2018). Thus, the present study aimed to adapt the *threshold model*, which claims that ECAs can promote academic and non-academic development as intended as long as the situation is optimal (Marsh and Kleitman, 2002, p. 472). The model suggests that students who invest too much time in extracurricular activities (including the Arts) may neglect schoolwork and, in turn, academic outcomes suffer. Some research supports this notion, finding diminishing returns and a reduction in academic performance due to intense extracurricular activity (Mansour, 2013). Marsh tested the assumption on the outcomes of twelfth and postsecondary students, revealing a linear and non-linear effect of participation in ECAs (Marsh, 1992). In China, children are under strict parental supervision that exhibits intensive demanding and pressing to make them flourish in academic and non-academic aspects; thus, parents are the ones who intensively follow their children’s out-of-school ECAs and academic time allocation based on China’s meritocracy (children’s future lives are strictly related to their academic performance).

## Materials and methods

### Participants

The present study conducted a cross-section survey research design in light of the paramount objective of the study. As we mentioned above, studies on visual art education in China, even as ECAs, have primarily been limited to economically well-off cities of China, which is an entirely inappropriate setting to investigate the effect of cultural capital and the application of ECAs. Therefore, we recruited a large randomized sample of 2,437 children (grades 1–6) between the ages of 7 and 14 (M = 12.6, SD = 2.03) to attempt the survey from 12 public primary schools that were randomly selected from public schools in Province Y, located in the southeastern part of China (see Table 1). Initially, before dispatching our questionnaire, the parents of 3,000 primary school children selected from all primary schools in the province were asked to return informed consent forms. After waiting for 2 weeks, we obtained consent from 2,861 parents for their children to participate in the study. Then, we dispatched a survey written in Mandarin for each grade level of sampled children with substantial support from teachers and head teachers. After collecting the paper-based questionnaires, we omitted 424 questionnaires that were unfinished or had missing or inappropriate responses, yielding a final dataset containing 2,437 responses.

RETRACTED

**TABLE 1:** Demographic information of the sample.

Variables	M (SD)%
Children age	12.6 (2.03)
Gender (Female)	852 (52.5%)
Percentage of only child	14.9%
Percentage of at least one parent migrant	53.3%
**Marital status**	
Married	80.1%
Divorce	10.5%
Remarried	7.2%
Widowed	2.2%
**Mother educational level**	
Didn’t finish primary school	13.1%
Primary School	21.4%
Junior high school	36.9%
Vocational High school	6.5%
Senior high school	15.2%
Undergraduate and above	6.8%
**Father educational level**	
Didn’t finish primary school	8.6%
Primary School	19.4%
Junior high school	40.0%
Vocational High school	7.4%
Senior high school	16.4%
Undergraduate and above	8.2%
**Mother monthly income**	
Under 1,000 RMB	28.8%
1,000–3,000 RMB	44.0%
3,000–6,000 RMB	20.6%
6,000–9,000 RMB	4.4%
Over 10,000 RMB	2.2%
**Father monthly income**	
Under 1,000 RMB	16.1%
1,000–3,000 RMB	40.4%
3,000–6,000 RMB	28.5%
6,000–9,000 RMB	11.0%
Over 10,000 RMB	4.0%

### Measurements

#### Socioeconomic status

The socioeconomic status of our participants was measured with two common indicators: parents’ educational levels and monthly income. Many studies have measured parental educational levels (father and mother) with 4- to 5-point Likert scales. However, the present study investigates a low-SES province in which the society exhibits a diverse range of parental educational attainment. Accordingly, parental educational level (for both fathers and mothers) was captured with the following 7-point Likert scale: 1 = did not finish elementary school (8.6% of fathers and 13.1% of mothers), 2 = completed primary school (21.4 and 19.4%, respectively), 3 = completed junior high school (36.9 and 40.0%, respectively), 4 = completed vocational high school (6.5 and 7.4%, respectively), 5 = completed regular senior high school (15.8 and 14.5%, respectively), 6 = completed junior college (15.2 and 17.4%, respectively) and 7 = completed a university undergraduate or postgraduate degree (6.8 and 8.2%, respectively).

RETRACTED

The distribution of parental educational levels confirms our speculation that rural Chinese parents’ educational levels are not normally distributed. The other SES indicator is monthly parental income, which was reported by each participating student’s parents or legal guardians (grandparents) on a five-point Likert scale: 1 = under 1,000 RMB, 2 = 1,000–3,000 RMB, 3 = 3,000–6,000 RMB, 4 = 6,000–9,000 RMB, and 5 = over 9,000 RMB.

#### Art participation

We designed 12 items that assess children’s participation in out-of-school art schools and visual arts activities. The items were rated on a 5-point Likert scale ranging from 1 = strongly disagree to 5 = strongly disagree. Sample items include “I often go to art exhibitions or community cultural activities,” “I like all kinds of courses related to art,” and “I draw many visual elements such as lines, shapes, spaces, and colors.” The Cronbach’s alpha coefficient value was 0.83.

#### Art interest

Ten items were included in the survey to measure children’s interest in or affection for visual art-related activities. The items were rated on a 5-point Likert scale ranging from 1 = strongly disagree to 5 = strongly disagree. Sample items include “I feel happy when I appreciate art works,” “I have a strong interest in the artistic emotion conveyed in film and television works and images,” and “I am good at discovering beautiful things in my life through observation.” The internal consistency reliability coefficient (Cronbach’s alpha) was 0.80.

#### Parental support

The involvement of parents in their children’s out-of-school visual art participation was comprehensively measured in this study by considering their time and financial investment to support their children’s art activities. The items were rated on a 5-point Likert scale ranging from 1 = strongly disagree to 5 = strongly disagree. Sample items included “My parents can understand the inner meaning of my works,” “My parents always support me to attend art-related training,” and “My parents often go to see exhibition halls, museums, and art galleries with me during holidays.” The Cronbach’s alpha coefficient value was 0.78.

RETRACTED

#### Academic performance

Given that the participants in the present study were elementary school students in grades 1 to 6, we could not use scores from standardized tests. Therefore, given that the final examinations vary with school and grade, we standardized all the test scores to eliminate the potential impact of school and grade. We standardized the Chinese, English, and math scores using the score distribution in the specific school and the student’s grade. All subsequent analyses utilized these standardized scores as the children’s test scores.

### Data analysis procedures

After collecting all the necessary data, the next task was to encode the student questionnaires that had no missing responses in SPSS 23.0. This analysis software was used to conduct descriptive, multivariate, and bivariate analyses to show the associations among the variables. Then, AMOS 21.0 was used to conduct SEM or path analysis to examine the size of the effect of multiple mediating variables and other direct and indirect effects. The mediating role of parental support is primarily considered for testing the threshold model by assuming parental support mediates the relationship between out-of-school visual art activity and academic performance.

### Research findings

Due to the nature of the variables measured, we conducted a two-way multiple analysis of covariance (MANCOVA) to inspect the effect of age and gender on children’s perceived art interest, participation, and parental support. Table 2 presents the MANCOVA results, which demonstrate a surprising finding that the end of primary school is the beginning of adolescence. The results indicate that art interest (*F* = 0.491, *P* = 0.484, η^2^ = 0.036), participation (*F* = 2.331, *P* = 0.127, η^2^ = 0.020), and parental support (*F* = 0.972, *P* = 0.324, η^2^ = 0.041) are not significantly different across 7- to 14-year-old primary school students. However, the MANCOVA findings showed a substantial difference in the perceived visual art interest (*F* = 49.016, *P* < 0.001, η^2^ = 0.170), participation (*F* = 35.813, *P* < 0.001, η^2^ = 0.220), and parental support (*F* = 12.794, *P* < 0.001, η^2^ = 0.195) of boys and girls.

**TABLE 2:** MANCOVA result of the operating variables.

	Gender							
	Boys		Girls		F	Age		F
	M	SD	M	SD		β	SE	
Art interest	3.080	0.799	3.295	0.709	49.016***	0.012	0.017	0.491
Art participation	2.881	1.023	3.124	0.984	35.813***	0.035	0.023	2.331
Parental support	2.795	1.213	2.973	1.237	12.794***	0.028	0.028	0.972

***p < 0.001.

Table 3 indicates the bivariate correlation among all variables regressed in the current study. SES (mothers’ and fathers’ educational levels and incomes) is positively correlated with student academic performance. According to the correlation results, fathers’ and mothers’ educational levels have a significant robust, strong, positive correlation with their monthly earnings (*r* = 0.813, *P* < 0.001 and *r* = 0.718, *P* < 0.001, respectively), which explains the Chinese meritocratic political system. Regarding out-of-school participation in visual arts, mothers’ educational levels (*r* = 0.580, *P* < 0.001) and monthly wages (*r* = 0.469, *P* < 0.001) had stronger associations than fathers’ education (*r* = 0.166, *P* < 0.001) and monthly income (*r* = 0.276, *P* < 0.001). Likewise, solid support comes from mothers who are educated (*r* = 0.654, *P* < 0.001) and have sufficient income (*r* = 0.562, *P* < 0.001). Most importantly, the bivariate analysis found that students’ perceived visual art participation impacted their school performance in Chinese (*r* = 0.570, *P* < 0.001), English (*r* = 0.794, *P* < 0.001), and math (*r* = 0.667, *P* < 0.001). Moreover, Table 3 shows that high achievers in Chinese (*r* = 0.791, *P* < 0.001), English (*r* = 0.596, *P* < 0.001), and math (*r* = 0.557, *P* < 0.001) showed a responsive interest in visual arts.

RETRACTED

**TABLE 3:** Bivariate correlation analysis.

	M	SD	α	1	2	3	4	5	6	7	8	9	10
FE	3.32	1.459	0.783	1									
FI	3.15	1.495	0.813	0.635	1								
ME	2.49	1.020	0.821	0.241	0.192	1							
MI	2.10	0.941	0.760	0.201	0.281	0.218	1						
Chinese	76.50	0.154	0.803	0.425	0.301	0.299	0.373	1					
English	79.81	0.320	0.751	0.345	0.333	0.326	0.307	0.751	1				
Math	77.57	0.457	0.830	0.463	0.333	0.323	0.430	0.438	0.629	1			
AI	3.1930	0.761	0.816	0.138	0.149	0.551	0.352	0.791	0.596	0.577	1		
ARP	3.0080	1.010	0.767	0.166	0.276	0.580	0.469	0.570	0.794	0.667	0.818	1	
PS	2.8884	1.229	0.810	0.235	0.358	0.654	0.562	0.010	0.092	0.139	0.611	0.600	1

All correlation values are significance < 0.001. FE, father education; FI, father monthly income; ME, mother education; MI, mother monthly income; AI, art interest; ARP, art participation; PS, parental support.

Structural equation model or path analysis was performed using AMOS 21.0 to examine the parallel and serial mediating role of the speculated variables. The results of the SEM indicate a good model fit. The chi-squared [χ^2^_(29)_ = 880.615], goodness-of-fit index (GFI, 0.97), the comparative fit index (CFI, 0.968), and mean square error of approximation (RMSEA, 0.005) values were highly significant (*P* < 0.001), which implies that the model fit the data well. Moreover, the model administered a bootstrap method to test the parallel and serial mediating role of art interest, parental support, and visual art participation in the relationship between socioeconomic status and academic performance over 5,000 samples. The parallel and serial mediating effect was significant, accounting for 38% of the variance. These findings confirmed our hypothesis (see Table 4).

RETRACTED

**TABLE 4:** Direct and indirect effects.

Indirect effect path	Mediators	Effect	95% CI
SES-PS-AP	Parental support	0.001	[–0.021, 0.018]
SES-ARP-AP	Art participation	0.002	[–0.031, 0.041]
SES-AI-AP	Art interest	0.03***	[0.041,0.001]
SES-PS-ARP-AP	Parental support and art participation	0.0003	[–0.010, 0.022]
SES-AI-PS-AP	Art interest and parental support	0.001	[–0.001, 0.0034]
SES-AI-ART-AP	Art interest and art participation	0.003	[–0.051, 0.073]
SES-AI-PS-ARP-AP	Art interest, parental support, and art participation	0.001	[0.0081, 0.0098]

No start = *p* < 0.001, *p < 0.01, **p < 0.05, ***not significance; AP, academic performance.

Further supporting the present study hypotheses, the SEM finding indicates that children’s active participation in visual art activities is significantly related to their interest in the activity (β = 0.68, *P* < 0.001), which verified our first hypothesis. Similarly, the serial model result confirms the present study’s second hypothesis that children’s art interest has an indirect effect on their active visual art participation through the mediating role of parental support (β = 0.11, *P* < 0.001). Unfortunately, the path analysis failed to accept the third hypothesis that children’s active visual art participation fosters their academic performance, given that the model showed that there is a substantial relationship between them (β = 0.03, *P* = 0.510). On the other hand, the path analysis result supports our fourth hypotheses, which further support socioeconomic status robustly affecting student academic performance (β = 0.24, *P* < 0.001), art interest (β = 0.16, *P* < 0.001), parental support (β = 0.06, *P* < 0.05), and active visual art participation (β = 0.07, *P* < 0.001). Regarding our fifth hypothesis, which stated that art interest, parental support, and visual art participation mediates the impact of SES on academic performance, the findings of the present study are partially supportive since the finding elucidates that except for art interest (β = 0.03, *P* < 0.001), SES does not have an indirect effect on academic performance through mediating the relationship between parental support (β = 0.001, *P* = 0.301) and visual art participation (β = 0.002, *P* = 0.740). Ultimately, the serial mediation model of the current study negates our last hypothesis that art interest, parental support, and visual art participation serially mediate the relationship of parental socioeconomic status and academic performance. However, the serial mediation model result indicates no significant serial mediating role of SES-AI-PS-AP (β = 0.001, *P* = 0.061), SES-AI-ARP-AP (β = 0.003, *P* = 0.093), SES-PS-ARP-AP (β = 0.0003, *P* = 0.757), or SES-AI-PS-ARP-AP (β = 0.001, *P* = 0.089) (Figure 1 and Table 4).

RETRACTED

**FIGURE 1:** Structural equation model analysis to test the threshold model. No start = *p* < 0.001, **p < 0.05, ***not significance; FE, father education; FI, father monthly income; ME, mother education; MI, mother monthly income; SES, socioeconomic status; AP, academic performance.

## Discussion

The present study used the threshold model to evaluate the effect of out-of-school visual art participation on children’s academic development through parents’ support in China, which is presumed to balance children’s ECAs and academic time (Marsh and Kleitman, 2002). Unfortunately, in contrast to the implications of the *threshold model*, the SEM findings showed that Chinese parental support does not affect the impact of out-of-school art participation on academic performance. The preliminary findings of this paper contradict a large body of evidence that stated that children lose interest in ECAs when they become teenagers or adolescents (Smith and Smith, 2008; Mansour et al., 2016; Foster and Marcus Jenkins, 2017; Jindal-Snape et al., 2018; Morris, 2018; Ye, 2018), although the findings are in line with a single study (Marsh and Kleitman, 2002). Existing evidence has shown that parents withdraw their children from ECAs they are interested in so that their children can focus on the university entrance examination that predicts their future life paths (Choi et al., 2005; Ho, 2011; Mansour et al., 2016; Qurban et al., 2019). However, such an explanation does not apply to our findings, given that the present study targeted primary school-age children and adolescents who are not old enough to engage in academic-related activities only due to national examinations.

In addition, parental support and children’s out-of-school visual art participation were uniforms throughout the data. A possible explanation for this finding is that those children who participate in out-of-school visual art activities do so due to their interest in the ECA, which allows them to maintain their interest and involvement as they grow. Fortunately, the MANCOVA results concur with previous studies that showed girls to be more interested in visual arts than boys (Anderson et al., 2003; McManus and Furnham, 2006; Smith and Smith, 2008; Mansour et al., 2016; Ye, 2018; Qurban et al., 2019; Kong, 2021) since boys feel that participating in activities that involve coloring, painting, and drawing is feminine. Moreover, the multivariate results indicate that Chinese parents provide more financial and time support for girls than boys, ensuring their parents’ art interests will be respected.

RETRACTED

The fundamental aim is to examine the direct and indirect effects of SES on academic performance through the serial mediation role of art interest, parental support, and out-of-school visual art activities in contemporary China that enable us to assess the linear and non-linear effect of out-of-school visual art activities through the lens of the threshold model. In the meantime, this allows us to determine the distinct mediating roles of art interest, parental support, and art participation in the relationship between SES and children’s academic attainment. According to the path model, SES has robust direct power to determine children’s academic achievement in contemporary China, providing substantial evidence internationally and in China (e.g., Covay and Carbonaro, 2010; Li and Qiu, 2018; Liu et al., 2020). However, recent Chinese studies have called for further investigation to understand the potential intervening variables that explain the association between SES and student academic attainment in more economically well-off provinces (Liu et al., 2020). This study contributes to the literature in the Chinese context by showing that the causal relationship between SES and learning outcomes is mediated by ECA participation (Covay and Carbonaro, 2010). Moreover, the present study considered not only the involvement of children in visual art activities but also the interest they possess and the support they obtain from their parents to guide the study using threshold theory (Marsh and Kleitman, 2002).

According to the model’s findings, affluent children are more likely to sustain interest in visual art activities, receive parental support, and actively participate in visual art activities. Expectedly, this finding supports many Chinese (Zhang and Tang, 2017; Ye, 2018; Ren et al., 2020) and Western studies that have shown that high family SES determines out-of-school ECAs (McManus and Furnham, 2006; Covay and Carbonaro, 2010; Kadar-Satat, 2015; Mansour et al., 2016; Foster and Marcus Jenkins, 2017; Morris, 2018). Plausibly, the study also reflects the Chinese parental culture in which mothers’ SES is a robust determinant of a child’s ECA involvement (Lau and Cheng, 2016; Zhang and Tang, 2017; Chiu and Lau, 2018; Kong, 2021). In addition to parents’ financial investments, studies have suggested that children require spending time in and out of the house with their parents to illuminate their ECA cognition (Ho, 2011; Morris, 2018; Ye, 2018; Qurban et al., 2019; Kong, 2021). Likewise, substantial evidence suggests that a high SES in China enables parents to provide more support and time for children’s ECA development than their low SES counterparts, which requires parents to spend their days working multiple jobs (Poon, 2020), which results in low SES children wasting their free time on non-beneficial or risky activities (Dumais, 2006). This proves that, in addition to educational outcomes, modern affluent parents show the value they have and support for their children’s out-of-school ECAs by spending time with their children during in and out-of-home activities, which contradicts the outdated perception of wealthy parents’ diligence (Ho, 2011; Gao et al., 2022). Simultaneously, the present study affirms that visual art, among all ECAs, requires a sincere interest, persistence, and affection from child participants (Lowry and Wolf, 1988), perhaps due to modern Chinese parental trust and respect for their children’s ECA interests (Zhang and Tang, 2017; Qurban et al., 2019), which contradicts the characterization of Chinese parenting as aggressive (Choi et al., 2005; Ho, 2011; Lau and Cheng, 2016; Chiu and Lau, 2018, p. 478; Poon, 2020). Instead, our study confirms our assumption that modern Chinese parents genuinely support their children’s active participation in their interest in ECAs. As a result, children’s art interests play the most significant role in determining their school performance and mediating the relationship between SES and academic performance. Likewise, an emerging body of evidence well-addressed that such intended outcomes can be obtained only when children have a definite interest in the specific activity and genuine support from their parents (Zhang and Tang, 2017; Qurban et al., 2019). Moreover, visual arts are unlike other ECAs require a genuine and persistent interest (Lowry and Wolf, 1988).

RETRACTED

Arguably, the current study found no relationship between children’s participation in visual art activities and academic attainment (Marsh and Kleitman, 2002; Foster and Marcus Jenkins, 2017). In view of Marsh and Kleitman’s explanation, children’s participation in out-of-school ECAs has a weaker influence on student school-related performance than in-school ECAs. A possible explanation is that the children may participate in several ECAs in addition to the visual art activities, which might adversely affect their academic work (Lau and Cheng, 2016). Additionally, another potential explanation was given by Mansour et al. (2016): high academic achievement students are interested in and participate in visual art activities in and out of school. Thus, our study argues that visual art activities promote positive academic performance as long as children participate in solely one out-of-school ECA, particularly a visual art program, which is more closely related to the academic development of children than other ECAs (Jolley and Zhang, 2012). Alternatively, our evidence noted that academically strong and affluent children with a strong interest in visual art activities do not need support from their parents or out-of-school visual art activities if they have the time management and art resources available at home. A study in China highlighted that children with a high SES do not benefit from out-of-school ECAs since they have easy access at home to polish their visual art skills (Ren et al., 2020).

These findings take us to the threshold theory that ECAs can promote academic and non-academic development as intended as long as the situation is at the optimal point (Marsh and Kleitman, 2002, p. 472). The model stated that children who invest excessive time in ECAs due to a lack of parental support exhibit worse academic achievement (Mansour, 2013). Consequently, the serial mediation model affirms that although children participate in visual art activities and are interested in robust parental support, active participation does not significantly promote their academic performance. Unfortunately, the study found that visual art participation has no significant impact on academic achievement, although its effect is greater for children whose sole ECA is art (Lowry and Wolf, 1988; Piscitelli et al., 1999; Chiu and Lau, 2018; Kong, 2021). Thus, this finding suggests that the advantage of being in ECAs is more prominent if parents consider their children’s interests. Concurrently, the results exposed the hidden power of SES in the era of compulsory Chinese education (Zhang and Tang, 2017; Li and Qiu, 2018; Ye, 2018; Liu et al., 2020; Ren et al., 2020), which results in educational inequity and inequality (Covay and Carbonaro, 2010; Kadar-Satat, 2015; Foster and Marcus Jenkins, 2017; Kong, 2021). Simultaneously, the serial mediation model provides unexpected results which show that in the Chinese context, parental support is unrelated to children’s art participation and enhancing their cognitive skills. An earlier article written by an art education scholar affirms that academically strong students are more likely to be involved in out-of-school extracurricular, particularly in visual arts; thus, if art participation does not affect academic performance at any time, it will not interrupt children’s schoolwork since outperforming students know how to manage their time (Mansour et al., 2016). Likewise, based on Chinese political philosophy, students are fully aware of the value of their academic performance in their future lives (Choi et al., 2005; Ho, 2011; Lau and Cheng, 2016; Chiu and Lau, 2018, p. 478; Poon, 2020), so it is unquestionable that Chinese students practice extensive self-control built from early childhood Confucian social adjustment (Lockette, 2012; Ho et al., 2017; Chiu and Lau, 2018; Qurban et al., 2019; Kong, 2021). This nuanced evidence explains why, unlike Western children, Chinese children have incredible self-control cultivated by the family, school, and society, enabling them to inhabit undesirable and maladaptive behavior that destructs their academic, social, and physical adjustments. Consequently, the model does not apply to Chinese and culturally related societies where children can waste time on ECAs without intensive parental support.

RETRACTED

## Conclusion

The present study sought to extend the Threshold model (Marsh and Kleitman, 2002), which suggests the application of ECAs in fostering positive academic performance up to a certain point; nevertheless, it may diminish children’s academic adjustment by virtue of excessive time pledge in ECAs (Seow and Pan, 2014). The preliminary finding of the study stipulates that in contemporary Chinese society, children’s interest in visual art, parental support for it, and the likelihood of participating in out-of-school visual art activities are determined by family SES. However, unexpectedly the current study finding suggested that children’s participation in out-of-school visual art activities doesn’t have a substantial value in promoting children’s academic performance in the face of genuine interest and supportive parenting, which negates the threshold model that was suited in a large body of western evidence. From the discussion of the present study finding and existing literature, it is plausible to conclude that academically high achievers practice robust time management skills without intensive parental supervision and guidance that would assist them in pursuing extracurricular arts in addition to their curricular commitments and responsibilities (Mansour et al., 2016), which initiate potential speculation that if students are interested and involve in visual art activities aside from other ECAs, the odd of those students’ success strong are exceedingly high. Moreover, in light of the study setting society cultural ideology, unlike Western child-rearing, Chinese children go through strict academically oriented parenting, rendering them independent of parental support and supervision to manage their academic time at a non-academic early age.

### Implications and limitations

This study has a robust policy and practical and theoretical implications for the future directions of in- and out-of-school visual art and other ECAs. The government of China should consider promoting visual art education in early childhood and primary education curricula to lay a solid foundation for self-esteem, self-concept, and self-efficacy skills that are critical for cognitive development and cannot be obtained at a later age since children will be busy with academic tasks to prepare for tertiary entrance examinations and to eliminate the dominant effect of SES on student academic performance. Furthermore, the government should encourage teachers who are well-trained and qualified to teach visual arts or, in the case of resource contain, to integrate visual arts comprehensively with other core subjects, such as science, technology, engineering, art, and math (STEAM), which supports the true purpose of visual arts for children. Moreover, the present study recommends that society, schools, and parents encourage boys to participate in visual art activities. For instance, instead of mothers, fathers are encouraged to become involved in visual art activities with their sons so that sons feel comfortable with the influence of their fathers. Theoretically, the model is more suitable for Western countries where children grow up with loose parental control, resulting in low self-control over their academic and non-academic time. However, more studies are still required to support such claims.

RETRACTED

Although this paper rigorously analyzed large-scale data, there are multiple limitations that the study could not address and should be considered by future studies. In this paper, only one of the 36 Chinese provinces was studied. It is inappropriate to generalize the findings to other provinces and countries. Therefore, Chinese and international scholars are encouraged to conduct more methodologically rigorous investigations of visual arts in provinces where little is known. Accordingly, quasi-experimental studies that compare the non-cognitive skills (self-esteem, self-efficacy, self-concept, and creativity) if children exposed to art activity and those not exposed to comparable schools are highly recommended. Our study did not measure parental support in detail by considering whether parenting support is aggressive or pressurized. Thus, future studies are advised to keep this in mind. Additionally, for future studies in China, young children familiar with visual arts can be identified to inspect the substantial effect of art education on their non-academic skills by involving parents and school aesthetic teachers.

## Data availability statement

The raw data supporting the conclusions of this article will be made available by the authors, without undue reservation.

RETRACTED

## Ethics statement

The studies involving human participants were reviewed and approved by Shenzhen University. Written informed consent to participate in this study was provided by the participants’ legal guardian/next of kin.

## Author contributions

SK and ET conceived and carried out the study, participated in its design, performed the statistical analysis, and drafted the manuscript. CG supervised the study, participated in the study’s design, helped to draft the manuscript by administering the survey in Mandarin language. ML critically revised the manuscript. All authors read and approved the final manuscript.

## References

[B1] AndersonJ. C.FunkJ. B.ElliottR.SmithP. H. (2003). Parental support and pressure and children’s extracurricular activities: Relationships with involvement and affective experience of participation. *J. Appl. Dev. Psychol.* 24 241–257. 10.1016/S0193-3973(03)00046-7

[B2] BourdieuP. (1973). The three forms of theoretical knowledge. *Soc. Sci. Inform.* 12, 53–80. 10.1177/053901847301200103

[B3] ChiuC. Y.LauE. Y. H. (2018). Extracurricular participation and young children’s outcomes in Hong Kong: Maternal involvement as a moderator. *Child. Youth Serv. Rev.* 88 476–485. 10.1016/j.childyouth.2018.03.051

[B4] ChoiA. L. Y.TseJ. C. Y.SoC. S. N.YeungA. S. (2005). Hong Kong Parents’ Perceptions of Benefits of Music to Their Children. *New Horiz. Educ.* 51 111–123. 32977785

[B5] CovayE.CarbonaroW. (2010). After the bell: Participation in extracurricular activities, classroom behavior, and academic achievement. *Soc. Educ.* 83 20–45. 10.1177/0038040709356565

[B6] DumaisS. A. (2006). Elementary School Students’ extracurricular Activities: The Effects of Participation on Achievement and Teachers’ evaluations. *Soc. Spectr.* 26 117–147. 10.1080/02732170500444593

[B7] FosterE. M.Marcus JenkinsJ. V. (2017). Does participation in music and performing arts influence child development?. *Am. Educ. Res. J.* 54 399–443. 10.3102/0002831217701830

[B8] GaoC.TadesseE.KhalidS. (2022). Family socioeconomic status and the parent–child relationship in Chinese adolescents: The multiple serial mediating roles of visual art activities. *BMC Public Health* 22:1018. 10.1186/s12889-022-13215-8 35596160PMC9123813

[B9] HoR. T.LaiA. H.LoP. H.NanJ. K.PonA. K. (2017). A strength-based arts and play support program for young survivors in post-quake China: Effects on self-efficacy, peer support, and anxiety. *J. Early Adolesc.* 37 805–824. 10.1177/0272431615624563

[B10] HoW. C. (2011). Parental support and student learning of musical instruments in Hong Kong. *Vis. Res. Music Educ.* 19:5.

RETRACTED

[B11] HuiA. N.HeM. W.YeS. S. (2015). Arts education and creativity enhancement in young children in Hong Kong. *Educ. Psychol.* 35 315–327. 10.1080/01443410.2013.875518

[B12] JinY. (2017). *A cross-cultural study of contemporary early childhood arts curricula.* Ph.D thesis, Australia: Flinders University, School of Education.

[B13] Jindal-SnapeD.DaviesD.ScottR.RobbA.MurrayC.HarkinsC. (2018). Impact of arts participation on children’s achievement:A systematic literature review. *Think. Skills Creat.* 29 59–70. 10.1016/j.tsc.2018.06.003

[B14] JolleyR.ZhangZ. (2012). How drawing is taught in Chinese infant schools. *Int. J. Art Design Educ.* 31 30–43. 10.1111/j.1476-8070.2012.01726.x

[B15] Kadar-SatatG. (2015). *Participation in out-of-school activities and the socioeconomic gap in children’s academic outcomes.* Ph.D thesis, Edinburgh: University of Edinburgh.

[B16] KongS. H. (2021). A study of students’ perceptions of parental influence on students’ musical instrument learning in Beijing. China. *Music Educ. Res.* 23 287–299. 10.1080/14613808.2020.1832978

[B17] LauE. Y. H.ChengD. P. W. (2016). An exploration of the participation of kindergarten-aged Hong Kong children in extra curricular activities. *J. Early Child. Res.* 14 294–309. 10.1177/1476718X14552873

[B18] LawW. W.HoW. C. (2011). Music education in China: In search of social harmony and Chinese nationalism. *Br. J. Music Educ.* 28 371–388. 10.1017/S0265051711000258

[B19] LiZ.QiuZ. (2018). How does family background affect children’s educational achievement? Evidence from Contemporary China. *J. Chin. Soc.* 5:13. 10.1186/s40711-018-0083-8

[B20] LiuJ.PengP.LuoL. (2020). The relation between family socioeconomic status and academic achievement in China: A meta-analysis. *Educ. Psychol. Rev.* 32 49–76. 10.1007/s10648-019-09494-0

[B21] LocketteK. F. (2012). Creativity and Chinese education reform. *Int. J. Glob. Educ.* 1, 2146–9296.

[B22] LowryK.WolfC. (1988). Arts education in the People’s Republic of China: Results of interviews with Chinese musicians and visual artists. *J. Aesthet. Educ.* 22 89–98. 10.2307/3332967

[B23] MansourM. (2013). *The role of school, home, and community Arts participation in students’ academic and non-academic outcomes.* Ph.D thesis, Australia: The University of Sydney.

[B24] MansourM.MartinA. J.AndersonM.GibsonR.LiemG. A. D.SudmalisD. (2016). Student, home, and school socio-demographic factors: Links to school, home, and community arts participation. *Aust. Educ. Res.* 43 221–244. 10.1007/s13384-015-0199-7

[B25] MarshH. W. (1992). Extracurricular activities: beneficial extension of the traditional curriculum or subversion of academic goals? *J. Educ. Psychol.* 84, 553–562. 10.1037/0022-0663.84.4.553

RETRACTED

[B26] MarshH.KleitmanS. (2002). Extracurricular school activities: The good, the bad, and the non-linear. *Harv. Educ. Rev.* 72 464–515. 10.17763/haer.72.4.051388703v7v7736

[B27] McManusI. C.FurnhamA. (2006). Aesthetic activities and aesthetic attitudes: Influences of education, background and personality on interest and involvement in the arts. *Br. J. Psychol.* 97 555–587. 10.1348/000712606X101088 17018189

[B28] MorrisJ. E. (2018). Arts engagement outside of school: Links with Year 10 to 12 students’ intrinsic motivation and self-efficacy in responding to art. *Aust. Educ. Res.* 45 455–472. 10.1007/s13384-018-0269-8

[B29] OECD (2016). *PISA 2015 Results (Volume I): Excellence and Equity in Education.* Paris: OECD Publishing. Available online at: 10.1787/9789264266490-en

[B30] PiscitelliB.Mai ChiP. T.ZhichaoC. (1999). Young children’s art education in Australia, Vietnam and China: A comparative perspective. *Asia Pac. J. Educ.* 19 21–30. 10.1080/0218879990190103

[B31] PoonK. (2020). The impact of socioeconomic status on parental factors in promoting academic achievement in Chinese children. *Int. J. Educ. Dev.* 75:102175. 10.1016/j.ijedudev.2020.102175

[B32] QurbanH.WangJ.SiddiqueH.MorrisT.QiaoZ. (2019). The mediating role of parental Support: The relation between sports participation, self-esteem, and motivation for sports among Chinese students. *Curr. Psychol.* 38 308–319. 10.1007/s12144-018-0016-3

[B33] RenL.ChenJ.LiX.WuH.FanJ.LiL. (2020). Extracurricular Activities and Chinese Children’s School Readiness: Who Benefits More? *Child Dev.* 92 1028–1047. 10.1111/cdev.13456 32840884

[B34] SeowP.-S.PanG. (2014). A Literature Review of the Impact of Extracurricular Activities Participation on Students’ Academic Performance. *J. Educ. Bus.* 89 361–366. 10.1080/08832323.2014.912195

[B35] SmithJ. K.SmithL. F. (2008). The structure of artistic and aesthetic abilities in school children. *Empir. Stud. Arts* 26 117–130. 10.2190/EM.26.1.h 22612255

[B36] YeW. (2018). Socioeconomic status and out-of-school citizenship education in China’s Shanghai. *Educ. Urban Soc.* 50 641–669. 10.1177/0013124517713609

[B37] ZhangD.TangX. (2017). The influence of extracurricular activities on middle school students’ science learning in China. *Int. J. Sci. Educ.* 39 1381–1402. 10.1080/09500693.2017.1332797

